The article "Ranibizumab for Macular Edema Secondary to Central and Branch Retinal Vein Occlusion in Patients Younger Than 50 Years of Age" was published in 2020. Journal: Biomed Res Int.

# Ranibizumab for Macular Edema Secondary to Central and Branch Retinal Vein Occlusion in Patients Younger Than 50 Years of Age

**DOI:** 10.1155/2020/4747696

**Published:** 2020-06-17

**Authors:** Maurizio Battaglia Parodi, Francesco Romano, Alessandro Arrigo, Stefano Mercuri, Alessandro Franceschi, Francesco Bandello

**Affiliations:** ^1^Department of Ophthalmology, University Vita-Salute, Scientific Institute San Raffaele, Milan, Italy; ^2^Eye Clinic, Department of Clinical and Biomedical Sciences, Luigi Sacco Hospital, University of Milan, Milan, Italy; ^3^Eye Clinic, Polytechnic University of Marche, Ancona, Italy

## Abstract

**Background:**

To determine the effectiveness of intravitreal ranibizumab (IVR) approach over 1-year follow-up in patients younger than 50 years old with central and branch retinal vein occlusion (RVO) complicated by macular edema (ME).

**Methods:**

Prospective, open-label case series. Patients initiating IVR injections from January 2015 to May 2017 were consecutively recruited. Each patient underwent monthly ophthalmic examination and structural OCT over 12 months. A single IVR injection was administered at baseline, followed by a PRN regimen. Outcome measures are best-corrected visual acuity (BCVA); central foveal thickness (CFT); number of IVR injections; subretinal fluid (SRF); epiretinal membrane; and outer retinal layer (ORL) status.

**Results:**

Thirty-eight patients (27 males) were included in the study. At follow-up, mean BCVA improved from 0.40 ± 0.17 to 0.10 ± 0.10 LogMAR in patients with central RVO and from 0.39 ± 0.19 to 0.19 ± 0.07 LogMAR in those with branch RVO, with 20 eyes gaining ≥3 ETDRS lines. In addition, mean CFT significantly decreased in both subgroups at the end of follow-up. All patients with SRF at baseline (9) disclosed complete resolution after 1 year. Likewise, ORL appeared reconstituted in most cases. At 12 months, 3.6 ± 2.4 and 4.4 ± 2.4 IVR injections were required for central and branch RVO, respectively, with only 5 eyes showing ME persistence.

**Conclusions:**

Our study indicates that IVR injections can be a valid therapeutic option in patients under 50 years of age with ME secondary to RVO.

## 1. Introduction

Retinal vein occlusion (RVO) in patients younger than 50 years of age represents a distinct subgroup of the disease, probably related to different pathogenetic mechanisms [1–6]. Possible complications occurring in this young population include macular edema (ME) and ocular neovascularizations [2–7]. Only a few studies have focused on the management of ME secondary to RVO in young adults [8, 9]. Overall, the natural history of this RVO subtype is believed to be more favourable with respect to older patients, as spontaneous improvement occurs in about one-fourth of cases in central RVO (CRVO) [10], with no specific study available instead for branch RVO (BRVO). Positive effects were shown by a single study based on dexamethasone implant in a subset of CRVO patients with best-corrected visual acuity (BCVA) better than 20/400 Snellen equivalents [11]. The aim of the current investigation is to improve the therapeutic approach to the disease, describing the clinical and morphological outcomes of therapy with intravitreal injections of ranibizumab (IVR) over 12 months of follow-up in patients younger than 50 years with ME secondary to CRVO and BRVO.

The article "Ranibizumab for Macular Edema Secondary to Central and Branch Retinal Vein Occlusion in Patients Younger Than 50 Years of Age" was published in 2020. Journal: Biomed Res Int.

## 2. Methods

The study was designed as a prospective, open-label, noncomparative case series. The investigation was approved by the local institutional review board and adhered to the tenets of the Declaration of Helsinki. Written informed consent was obtained from all the patients after complete explanation regarding the purpose of the study.

All patients younger than 50 years of age affected by RVO were prospectively recruited from January 2015 to May 2017. Inclusion criteria were as follows: (1) diagnosis of both CRVO and BRVO (patients younger than 50 years) with no previous treatment; (2) diagnosis of ME with central foveal thickness (CFT) ≥ 300 *μ*m on spectral-domain optical coherence tomography (SD-OCT) (Spectralis HRA+OCT; Heidelberg Engineering, Heidelberg, Germany); and (3) BCVA between 1.0 LogMAR (corresponding approximately to 20/200 Snellen equivalent) and 0.1 LogMAR (corresponding approximately to 20/25 Snellen equivalent). On the other hand, exclusion criteria included (1) any other ocular disorder able to confound the clinical assessment; (2) history of acute coronary event or stroke in the previous 6 months; (3) pregnancy or lactation; (4) any sign of ocular infection; and (5) presence of media opacities.

Each patient underwent an ophthalmic examination, including BCVA on standard Early Treatment for Diabetic Retinopathy Study (ETDRS) chart, anterior segment slit-lamp examination, Goldmann applanation tonometry, dilated fundus biomicroscopy, and fluorescein angiography using ultrawide-field angiography (UWF-FA; California®, Optos plc.). Ischemic CRVO was defined as the extension of capillary nonperfusion of at least 10 disc areas, whereas ischemic BRVO corresponded to capillary nonperfusion extension of at least 5 disc diameters [12, 13]. Fluorescein angiography could be repeated over the follow-up at examiner's discretion. A single intravitreal ranibizumab was administered at baseline, following a pro re nata treatment regimen based on monthly examinations. Further intravitreal ranibizumab injection was performed on the basis of the detection of intraretinal cysts and/or subretinal fluid on SD-OCT. BCVA measurement and SD-OCT scans were performed by masked ophthalmologists with regard to the patients' condition. The presence of subretinal fluid (SRF), epiretinal membrane (ERM), or any alteration of the outer retinal layers (namely, external limiting membrane (ELM); ellipsoid zone (EZ); and retinal pigmented epithelium (RPE)) was analysed both at baseline and at the end of follow-up. In particular, the condition of each layer within the foveal area was classified as either preserved (identification of a regular layer), disrupted (layer disorganization), or absent (loss of the layer).

The article "Ranibizumab for Macular Edema Secondary to Central and Branch Retinal Vein Occlusion in Patients Younger Than 50 Years of Age" was published in 2020. Journal: Biomed Res Int.

The primary outcome was to study the effectiveness of ranibizumab treatment assessing changes in BCVA at the end of the 12-month follow-up. Secondary outcomes included the correlations with the change in CFT and with the number of IVR injections over 12 months.

Shapiro-Wilk test was used to check the assumption of normality of the variables, while statistical analysis was performed by means of Wilcoxon test to evaluate the changes in BCVA and CFT. Results were expressed as mean ± SD for quantitative variables and as frequency (%) for categorical variables. All the analyses were performed using SPSS Statistics Version 23.0 Software package (IBM; Armonk, NY); all tests were two-tailed, and the level of significance was taken at *p* < 0.05.

## 3. Results

Overall, thirty-eight eyes of 38 patients were enrolled in the study, 25 being affected by CRVO and 13 by BRVO. The mean age was 41.7 ± 8.5 (range: 18-49 years) with 27 males (71%). The mean duration of RVO (calculated by the onset of symptoms as referred by patients) was of 9.4 ± 2.3 months, whereas the mean duration of ME (calculated by the first injection administered) was of 7.8 ± 1.6 months. Twenty-three patients (60.5%) were found to be hypertensive on therapy, 8 of them (21.1%) suffered from diabetes mellitus, and 3 (7.9%) were also affected by hyperlipidaemia. No patient turned out to be affected by coagulation or thrombophilic disorders. All patients complained of persistent visual disturbances and referred no subjective visual improvement over the 8 months of ME observation. UWF-FA revealed that all the patients with CRVO were affected by a nonischemic form of the disease, with no patient converting into ischemic CRVO over the follow-up. Differently, 4 patients with BRVO were affected by an ischemic subtype. All the patients attended the monthly scheduled visits and completed the 12 months of follow-up.

Taking into consideration patients affected by CRVO, the mean BCVA was 0.40 ± 0.17 LogMAR (range: 0.1-0.7 LogMAR) (approximately corresponding to 20/50 Snellen equivalent) at baseline, changing to 0.10 ± 0.10 LogMAR (0-0.3 LogMAR) (approximately corresponding to 20/25 Snellen equivalent) with a statistically significant improvement (*p* < 0.001). Looking at patients with BRVO, the mean baseline BCVA was 0.39 ± 0.19 LogMAR (range: 0.1-0.6 LogMAR) (approximately corresponding to 20/50 Snellen equivalent); after one year, the mean BCVA statistically improved up to 0.19 ± 0.07 LogMAR (range: 0-0.5 LogMAR) (approximately corresponding to 20/30 Snellen equivalent) (*p* < 0.01).  Table 1 illustrates the complete clinical and demographic data. At the end of the follow-up, the mean change from baseline BCVA letter score was of 15.1 ± 8.0 ETDRS letters for CRVO patients and of 7.0 ± 7.1 letters for BRVO patients. Fourteen of the 25 eyes (56%) with CRVO and 6 eyes (43%) with BRVO gained 3 or more ETDRS lines, whereas no eye lost 3 lines at the 12-month examination. Seventeen eyes (45%) achieved a BCVA of 0 LogMAR (approximately corresponding to 20/20 Snellen equivalent) at the end of the follow-up.

The article "Ranibizumab for Macular Edema Secondary to Central and Branch Retinal Vein Occlusion in Patients Younger Than 50 Years of Age" was published in 2020. Journal: Biomed Res Int.

In CRVO eyes, the mean CFT was 464 ± 211 *μ*m (range: 305-940 *μ*m) at baseline and 262 ± 69 *μ*m (range: 230-540 *μ*m) at the end of the follow-up, with a statistically significant difference (*p* < 0.001) (Table 1). Moreover, 12 eyes (48%) showed a CFT value within 300 *μ*m at the end of the study. On the other hand, examining eyes with BRVO, the mean CFT significantly decreased from 361 ± 80 *μ*m (range: 308-580 *μ*m) to 285 ± 57 *μ*m (range: 221-357 *μ*m) (*p* < 0.01).  Figure 1 shows the BCVA and CFT variations over the follow-up period.

In addition, although nine patients (24%) presented SRF at baseline, complete resolution was noticed in all the cases at the end of follow-up. Three patients (8%) disclosed ERM at baseline, with no change over the follow-up. Outer retinal layers were found to be thoroughly disrupted at baseline examination; however, at follow-up, these layers appeared reconstituted in the majority of cases, with ELM, EZ, and RPE remaining disrupted in fourteen eyes (37%). Graphic and SD-OCT representations of the main SD-OCT findings in CRVO and BRVO are reported in Figure 2.

Patients with CRVO received a mean of 3.6 ± 2.4 ranibizumab injections over the follow-up (range: 1-9), with four patients (16%) requiring only one injection and another four patients (16%) two injections. With regard to patients affected by BRVO, 4.4 ± 2.4 injections were required, with four eyes undergoing only one or two injections. At the end of the follow-up, 3 eyes with CRVO (12%) and 2 with BRVO (15%) showed persistence of ME, requiring further reinjections. No correlation was found between outer retinal layer conditions and visual outcome, as well as the number of injections. An exemplary case is shown in Figure 3.

The article "Ranibizumab for Macular Edema Secondary to Central and Branch Retinal Vein Occlusion in Patients Younger Than 50 Years of Age" was published in 2020. Journal: Biomed Res Int.

At the end of follow-up, no ocular or systemic side effects were registered nor ocular neovascularization developed over the follow-up.

## 4. Discussion

Retinal vein occlusion in patients younger than 50 years has been poorly investigated. Even though no precise information is available regarding the prevalence, the Beaver Dam study highlights a prevalence of 0.1 and 0.2% in CRVO and BRVO, respectively, in the age range between 43 and 54 years [14]. Overall, this subtype of RVO is generally considered to be characterized by milder clinical course [1–11]. The natural history is partially known only in patients affected by CRVO, but no information is available regarding BRVO course. A recent survey on CRVO reported a spontaneous BCVA improvement or decline of at least 3 lines in 23% and in 28% of the cases over the follow-up, respectively [10–19]. Several treatment options have been advocated including grid laser photocoagulation and intravitreal injections of corticosteroids and anti-VEGF molecules [8–12, 20–22]. In particular, only one previous investigation has specifically focused on CRVO in patients younger than 50 years of age, showing that intravitreal dexamethasone implants can be used to achieve significant functional improvement, with a visual gain of 3 or more lines in 50% of cases over 12 months [11]. However, about one-third of patients developed intraocular pressure elevation after dexamethasone implant. In addition, many patients are reluctant with respect to a potential treatment with dexamethasone implant in the fear of early cataract development. The alternative approach scheduling anti-VEGF injections in RVO patients younger than 50 was not explicitly analysed, even though all clinical trials included patients older than 18 years [23–28]. For these reasons, we decided to carry out a prospective and interventional pilot study to assess the effects of IVR for the management of ME in patients younger than 50 years affected by RVO.

Overall, BCVA significantly improved at the end of follow-up, with more than 50% of patients with CRVO and 43% with BRVO gaining at least 3 ETDRS lines and with a mean score gain of 15 and 7 letters, respectively. Likewise, the mean CFT was significantly reduced, with about half of the eyes achieving a CFT under 300 *μ*m. It is noteworthy that in our study, patients affected by BRVO seem to have less favourable visual outcomes with respect to CRVO, owing to the presence of four patients in the BRVO group with the ischemic form of the disease which showed limited functional and structural recovery. It seems difficult to compare our results with those from the CRUISE and BRAVO trials, as the inclusion criteria of the patients, regarding BCVA and CFT, were certainly different at baseline (worse BCVA, larger CFT, and exclusion of ischemic cases) with respect to our study [23–25]. However, this finding might further support the relative benign course of RVO in younger individuals. Similarly, different patients' inclusion criteria do not allow for comparison with the previous experience using intravitreal dexamethasone implant in patients younger than 50 years [11]. In order to expand the therapeutic applications, our study included also eyes with higher BCVA at baseline in the attempt to promote an optimal functional recovery in eyes affected by ME. Our study was based on a single IVR injection at baseline, followed by further injections on PRN regimen.

The article "Ranibizumab for Macular Edema Secondary to Central and Branch Retinal Vein Occlusion in Patients Younger Than 50 Years of Age" was published in 2020. Journal: Biomed Res Int.

Looking at the modifications of the outer retinal layers on SD-OCT, our data confirm the different patterns of layer reconstitution seen in this age subgroup with respect to that registered in older patients [29]. No correlation was found between SD-OCT patterns of the outer retinal layers and both the functional outcomes and the global number of injections at the end of follow-up, this possibly implying a different individual response to the anti-VEGF treatment, which cannot be predicted a priori using the current imaging tools. Maybe, genetic profiling along with baseline vessel density analysis and an in-depth investigation of the underlying pathogenetic causes might represent useful biomarkers to assess activity and severity of the disease.

We are aware that the present study has several limitations, especially including the limited number of patients, the shortness of the follow-up, and the absence of a control group. However, RVO represents a relatively infrequent condition in young adults and, thus, it is very difficult to design and plan a randomized clinical trial. Another important issue is related to the possible ceiling effect, particularly evident in BRVO, as several patients disclosed high BCVA at baseline and, therefore, could not achieve a significant gain in BCVA at 12-month follow-up. In addition, the delay of more than 7 months in treating ME, probably due to the relatively good visual function in this RVO subtype and the problems connected to the waiting list, may have limited the visual acuity gain. Furthermore, no control arm was present in order to compare the effect of the treatment; however, all our patients did complain of prolonged visual disturbances with persistence of ME for at least 7 months. Therefore, bearing in mind the young age of our cohort, corresponding to working age, we felt it is unethical to further delay or not offer at all a treatment for ME to these patients.

The article "Ranibizumab for Macular Edema Secondary to Central and Branch Retinal Vein Occlusion in Patients Younger Than 50 Years of Age" was published in 2020. Journal: Biomed Res Int.

In addition, we have to acknowledge that no patient in our series was affected by the ischemic form of CRVO; this finding might be the consequence of a more benign course of the disease in such a young population and might have positively affected visual and anatomical outcomes in this subgroup. For these reasons, no conclusion can be drawn at the moment regarding the best therapeutic strategy to approach ME secondary to RVO in patients younger than 50 years. In particular, we believe that both dexamethasone implant and IVR injections can be considered beneficial, and the therapeutic choice should probably rely on the comprehensive evaluation of many factors, including also patients' compliance and other systemic or ocular conditions.

## 5. Conclusion

In essence, the present investigation can be considered a pilot study indicating that a simplified IVR approach based on a single initial injection, followed by a PRN regimen, is a valid therapeutic option in patients younger than 50 years affected by ME secondary to RVO over a 12-month follow-up. Further studies are warranted in order to confirm our preliminary data.

## Figures and Tables

**Figure 1:** Mean visual acuity (in LogMAR) and central foveal thickness (in *μ*m) variations from baseline to the end of follow-up in patients with central (CRVO (a, b)) and branch retinal vein occlusion (BRVO (c, d)). Legend: LogMAR: logarithm of the minimal angle of resolution; FU: follow-up.

**Figure 2:** Graphic representation of the main optical coherence tomography findings at baseline and at 12-month follow-up in central (CRVO (a, b)) and branch retinal vein occlusion (BRVO (c, d)). Legend: SRF: subretinal fluid; ERM: epiretinal membrane; ELM: external limiting membrane; EZ: ellipsoid zone; RPE: retinal pigment epithelium.

**Figure 3:** Optical coherence tomography structural scan of a 34-year-old patient with macular edema secondary to central retinal vein occlusion. The scan in (a) shows the onset of the typical cystoid macular edema, complicated with subretinal fluid and disruption of the outer retinal layers. At 12-month follow-up (b), the edema appears resolved with restoration of the normal foveal anatomy and with a significant improvement in visual acuity, from 20/50 to 20/20 Snellen equivalents. Outer retinal layers turn out to be reconstituted.

**Table 1:** Clinical and demographic characteristics of eyes affected by central and branch retinal vein occlusion in patients aged under 50 years of age.

	All patients (*n* = 38)	Central RVO^∗^ (*n* = 25)	Branch RVO (*n* = 13)
Age (range)	41.7 ± 8.5 (18-49)	39.0 ± 9.6 (18-48)	43.4 ± 3.7 (28-49)
Sex (%)			
Male	27 (71%)	17 (68%)	10 (77%)
Female	11 (29%)	8 (32%)	3 (23%)
Baseline BCVA^†^ (range)		0.40 ± 0.17 LogMAR^‡^ (0.1-0.7)	0.39 ± 0.19 LogMAR (0.1-0.6)
(Snellen equivalents)		(20/50)	(20/50)
Follow-up BCVA (range)		0.10 ± 0.10 LogMAR (0-0.3)	0.19 ± 0.07 LogMAR (0-0.5)
(Snellen equivalents)		(20/25)	(20/30)
Baseline CFT^§^ (range)		464 ± 211 *μ*m (305-940)	361 ± 80 *μ*m (308-580)
Follow-up CFT (range)		262 ± 69 *μ*m (230-540)	285 ± 57 *μ*m (221-357)
Injections (range)		3.6 ± 2.4	4.4 ± 2.4

^∗^RVO: retinal vein occlusion. ^†^BCVA: best-corrected visual acuity. ^‡^LogMAR: logarithm of the minimal angle of resolution. ^§^CFT: central foveal thickness.

The article "Ranibizumab for Macular Edema Secondary to Central and Branch Retinal Vein Occlusion in Patients Younger Than 50 Years of Age" was published in 2020. Journal: Biomed Res Int.

## Data Availability

The data that support the findings of this study are available upon reasonable request from the corresponding author. Data requests should be made to Doctor Stefano Mercuri, mercuristef@gmail.com
